The article "Analysis of the Effectiveness of Transradial Access Puncture in the Application of Complications and Comfort after Cerebral Angiography" was retracted in 2023. Reasons: signs of a paper mill; compromised peer review; unreliable results or conclusions.

# Analysis of the Effectiveness of Transradial Access Puncture in the Application of Complications and Comfort after Cerebral Angiography

**DOI:** 10.1155/2022/3457034

**Published:** 2022-10-11

**Authors:** Hongyan Wan, Lan Gao, Daohua Huang

**Affiliations:** ^1^Zhongda Hospital Southeast University, Department of Interventional Radiology and Vascular Surgery, Nanjing 210009, China; ^2^Zhongda Hospital Southeast University, Department of Nursing, Nanjing 210009, China

## Abstract

**Objective:**

To investigate the analysis of the effectiveness of transradial access puncture in the application of complications and comfort after cerebral angiography.

**Methods:**

Retrospectively analyzed 80 patients who met the inclusion and exclusion criteria and were randomly divided into the control group (femoral artery group *n* = 40) and test group (radial artery group *n* = 40) using a random number table from January 2021 to January 2022 admitted to the department of neurology and department of vascular interventions in our hospital and compared the incidence of postoperative puncture site bleeding, time to first postoperative urination, and incidence of postoperative urinary retention and postoperative changes in comfort level.

**Results:**

There was 1 case of postoperative puncture site bleeding in the test group and 6 cases of postoperative puncture site bleeding in the control group, with statistically significant differences (*P* < 0.05); the time to first urination in the test group (62.47) was significantly better than that in the control group (85.97), with statistically significant differences (*P* < 0.05); there were 0 cases of urinary retention in the test group and 6 cases in the control group, with statistically significant differences (*P* < 0.05). The GCQ scores of patients in the test group were significantly higher than those in the control group, and the difference was statistically significant (*P* < 0.05).

**Conclusion:**

Transradial access puncture has a good clinical effect and can effectively reduce the complication rate of patients, which is worth promoting.

## 1. Introduction

In recent years, the incidence of various cerebrovascular diseases has shown a significant increase as the aging population in China continues to increase, and the main clinical symptoms of these diseases are distorted eyes and mouth and speech dysfunction, which seriously threaten the physical and mental health and quality of life of the elderly population due to the high disability and mortality rates [1]. Digital silhouette whole brain angiography and interventional therapy have been widely used in clinical medicine because of the advantages of convenient and simple operation and significant effect [2]. However, in the process of patient treatment, postoperative complications are likely to occur, which not only affect the effectiveness of treatment but also threaten the physical health of patients [3]. Therefore, effective measures must be taken to deal with the complications that occur in patients promptly.

The femoral artery itself has the advantages of coarse vessel diameter, relatively superficial location, clearer body projection, and high success rate of cannulation and is often used as the preferred channel for puncturing cerebral angiography, but is prone to puncture-related complications [4]. A study [5] counted 100 DSA inpatients and found that the incidence of vascular complications in patients with transfemoral access was 9.6%. The study [6] found that compression of the puncture site for 6 h was often required after transfemoral access puncture, and the operated limb also required 6–8 h of braking and 24 hours of bed rest. The study [7] found that prolonged postoperative bed rest is prone to many adverse effects, such as lumbar pain and discomfort, urinary retention, insomnia, and anxiety, which affect the postoperative recovery of patients to a greater extent.

The radial artery is relatively shallowly located, and the percutaneous radial artery vascular access test was first applied to coronary angiography in 1989 and first applied to interventional treatment in 1993 [8]. After years of practice, improvement, and refinement, transradial artery puncture has been gradually applied to cerebrovascular interventions [9]. The study [10] reported that the success rate of neurointerventional procedures with transradial access reached 94.5%, and the complication rate was also lower compared with transfemoral access puncture, which was only 2.9%. After transradial artery puncture, the puncture site requires compression bandaging, except for the wrist joint on the punctured side, which requires 6–8 hours of braking. The rest of the limb joints are not restricted in postoperative activities and have a high level of safety and comfort [11]. The study [12] showed that patients with transradial access usually had significantly less time in bed relative to 24 h after femoral artery surgery by 1.9.

Based on this, 80 patients who were admitted to the department of neurology and interventional vascular surgery from January 2021 to January 2022 and met the inclusion and exclusion criteria were selected for this study and randomly divided into a control group (femoral artery group *n* = 40) and a test group (radial artery group *n* = 40) using a random number table to compare the incidence of postoperative puncture site bleeding, time to first postoperative urination, and incidence of postoperative urinary retention in both groups. The results of the study were presented. The aim was to investigate the effectiveness of transfemoral and transradial arteries in terms of postoperative complications and comfort after cerebral angiography.

## 2. Objects and Methods

### 2.1. Object

Eighty patients who were hospitalized in our neurology and interventional vascular surgery departments from January 2021 to January 2022 and met the inclusion and exclusion criteria were selected, and the patients were randomly divided into a control group (femoral artery group, *n* = 40 cases) and a test group (radial artery group, *n* = 40 cases) using a random number table, with 16 females and 24 males in the control group, with a mean age of 62.679.44 years; in the test group, there were 20 female and 20 male cases with a mean age of 63.758.51 years. The study protocol was reported to and approved by the ethics department of our hospital before the trial, and the patients or their families were informed of the detailed study protocol and signed an informed consent form before the trial began.

#### 2.1.1. Inclusion Criteria

The inclusion criteria were as follows: history of cerebral ischemic or hemorrhagic cerebrovascular disease, cerebral aneurysm; suspicion of intracranial and extracranial arterial occlusion or stenosis, cerebral aneurysm by relevant MRA, CTA, carotid ultrasound, TCD, and other auxiliary examinations; negative Allen test results; good pulsation of the distal radial artery by transvascular ultrasound; conscious patients who can express themselves correctly; and patients who are unwilling to undergo femoral artery puncture.

#### 2.1.2. Exclusion Criteria

The exclusion criteria were as follows: patients who have used the radial artery for hemodialysis or other purposes; patients with arterial stenosis or lesions at the end of the hand; trauma to the hand or history of previous surgery; abnormalities in the vessels of the arm; and unwillingness to participate in this study.

### 2.2. Research Methodology

#### 2.2.1. Control Group

Patients underwent cerebral angiography with femoral artery access, and postoperative puncture sites were given inguinal pressure bandages (manufacturing license number: Su Food and Drug Administration Machinery Manufacturing Xu 20160050) for cross-row bandaging, and all patients were bandaged by the same physician. After the operation, the doctor and nurse in charge of the patient gave bedside instructions, instructed precautions and physical activities, applied local pressure and bandages to the puncture site of the operated limb for 6 h, and applied brakes for 6–8 h to keep the patient's hip joint straight. At the same time, the patient was instructed to perform an ankle pump exercise or massage the punctured side of the limb once every 2 hours.

#### 2.2.2. Test Group

Patients underwent cerebral angiography via radial artery access (TRA) puncture, and postoperative puncture sites were given elastic bandages (manufacturing license number: State Armament No. 20170241) for circumferential bandaging, and all patients were bandaged by the same physician. After returning to the ward after the operation, the doctor and nurse in charge of this patient performed bedside preaching, instructed precautions and physical activity patterns, local pressure bandaging of the punctured limb on the operation side for 6–8 hours, wrist braking for 6 hours, and unrestricted joints of the other limbs for 2 hours in bed.

#### 2.2.3. Postoperative Care Measures for Appropriate Complications

(1) Subcutaneous hematoma: The most common postoperative complication is mainly due to factors such as improper hemostatic methods or the patient's coagulation dysfunction. In addition to closely monitoring the patient's heart rate and blood pressure, the patient should be promptly and effectively treated for the tightness of the dressing, and the patient should be instructed to do effective care in daily life to avoid unnecessary bleeding. (2) Arterial thrombosis: Once the patient has a lower extremity temperature drop, numbness, pain, and other conditions, the possibility of arterial thrombosis is higher. Therefore, care should be taken to maintain the appropriate tightness of the bandage and closely monitor the color and temperature of the patient's limbs to effectively avoid the appearance of arterial thrombosis. (3) Urinary retention: A common complication is mainly caused by factors such as sudden changes in living habits or changes in emotions. Should pay attention to helping patients relieve bad psychological emotions in a timely manner and guide patients to carry out effective measures such as bed urination to help them deal with urinary retention in a timely manner.

### 2.3. Evaluation Indexes

#### 2.3.1. Incidence of Postoperative Puncture Site Bleeding

Incidence of postoperative puncture point bleeding = total number of cases of postoperative puncture point bleeding/total number of postoperative cases (40) × 100%. Postoperative puncture site bleeding can be divided into the following four conditions: (1) local bruising at the puncture site, mainly manifested as skin bruising with or without hard nodules around the puncture site; (2) local bleeding at the puncture site, manifested as blood oozing from the puncture site, around the balloon compression pad or on the dressing; (3) local hematoma at the puncture site, visible to the naked eye or local palpable hard nodules at the puncture site with a diameter >5 cm; (4) DSA and ultrasound imaging data in the presence of pseudoaneurysm are preferable.

#### 2.3.2. Time to First Postoperative Voiding and Incidence of Urinary Retention

Time of first urination refers to the time of first urination starting after the patient returns to the ward after surgery; urinary retention refers to the accumulation of a large amount of urine in the bladder that cannot be excreted by itself, which is mainly based on the patient's complaints and the doctor's percussion to initially determine whether urinary retention has occurred, and then determined by bedside ultrasonography.

#### 2.3.3. Changes in Postoperative Comfort

The General Comfort Questionnaire (GCQ) was developed by Kolcabas, an American comfort care specialist, to assess patients' comfort in postoperative bed rest, and consists of 4 physical, psychospiritual, environmental, and sociocultural dimensions and 28 items. The scale uses a Likert scale from 1 to 4, with 1 being “strongly disagree” and 4 being “strongly agree.” The higher the total score obtained, the higher the comfort level obtained by the patient. In 2006, the study [13] translated the scale into Chinese and tested its reliability, adding 2 items to the sociocultural dimensions to form a 30-item Chinese version of the GCQ. The Cronbach content of the Chinese version of the GCQ was also validated, with a validity of 0.86 and a coefficient of 0.92, which has high reliability and validity [14].

### 2.4. Efficacy Criteria

Use the homemade nursing satisfaction questionnaire to investigate the patient's satisfaction with nursing care using a self-made nursing satisfaction questionnaire, and the score is a percentage system. The higher the score, the higher the degree of satisfaction.

### 2.5. Data Collection

In accordance with the study design and process, study-trained, permanent staff conducted an informed script with patients who met the criteria and collected the required information after obtaining consent.

### 2.6. Statistical Methods

The collected data were entered into Excel by the double entry method, and then, the data in Excel were imported into SAS version 9.4 software for statistical analysis. The measurement data in this study were expressed as mean ± standard deviation, and the comparison of relevant data between groups was analyzed by the *t*-test, and the *P* < 0.05 between the two groups was statistically significant.

## 3. Results

### 3.1. Comparison of General Information between the Two Groups

During the implementation of this study, there were no lost cases or dropped cases in both groups, and there was no statistically significant comparison between the two groups in terms of general information (*P* > 0.05) (Table 1).

### 3.2. Comparison of Each Other Evaluation Index between the Two Groups

#### 3.2.1. Comparison of Postoperative Puncture Site Bleeding, Time to First Voiding, Urinary Retention, and GCQ

The (Table 2) incidence of complications in the two groups was significantly lower in the observation group than in the control group, and the data comparison was statistically significant (*P* < 0.05), as given in Table 2.

### 3.3. Nursing Satisfaction Statistics of Patients in Both Groups

The nursing satisfaction statistics of patients in the control group was 70.00% (28/40), which was much lower than the nursing satisfaction of 95.00% (38/40) of patients in the observation group, and the empirical evidence was statistically significant (*χ*^2^ = 9.680, *P* < 0.05).

## 4. Discussion

Cerebrovascular diseases, including cerebral atherosclerosis, cerebral artery injury, cerebral aneurysm, and cerebral arteriovenous fistula, account for 25–50% of neurological hospitalizations. DSA is the gold standard for the diagnosis of cerebrovascular disease and the basis for neurointerventional treatment, and specialized care with evidence-based medicine is increasingly important [15]. In this retrospective case-control study, the compliance rate of patients in the control group with high procedural compliance was lower than that in the intervention group, and the compliance rate of patients with low compliance was higher than that in the intervention group. The differences were statistically significant.

### 4.1. TRA Performed Cerebral Angiography Reduces the Rate of Bleeding at the Puncture Site

The study [15] reported that “radial artery occlusion and spasm, bleeding and hematoma, and vagal reflexes may occur after neurointerventional treatment of TRA.” The results of this study showed that the incidence of bleeding at the puncture site via TRA in the test group was 2.5% (1 case), but there were no complications such as radial artery spasm and occlusion and vagal reflexes, which is similar to the low incidence of complications (2.9%) of neurointerventional treatment via TRA in the study of the literature [7]. The incidence of puncture site bleeding was 12.5% lower in the trial group compared to the control group, and the difference between the two groups was statistically significant, with *P* values < 0.05 in both groups. However, *P* values > 0.05 for prothrombin time, platelets, and procedure time were not statistically significant in both groups. In addition, the TRA route has requirements for the surgeon and needs to be performed by a physician with some experience in the intervention and mastery of the technique.

### 4.2. TRA Cerebral Angiography Can Reduce the Incidence of Postoperative Urinary Retention

After transcatheter femoral artery puncture, patients are required to lie flat and the surgical limb is braked. A large proportion of patients have urinary retention due to various reasons such as long-term bed rest without changing position, pain at the puncture site, fear of bleeding from the puncture site, more unaccustomed to urination in bed, and anxiety and tension. After transcatheter radial artery puncture, local pressure dressing for 6–8 h, wrist braking for 6 h, and other limb joints of the extremities are not restricted, the time to get out of bed is 2 h later. This is similar to the results of the literature [16, 17] in which cerebral angiography through TRA was performed with a time to get out of the bed of 1.9. The shortened bedtime eliminated patients' concerns about bleeding at the puncture site and relieved their anxiety and tension, thus shortening the time to first postoperative urination and reducing the occurrence of urinary retention to a greater extent. In this study, the time to first postoperative urination was significantly better in the test group patients (62.47) than in the control group patients (85.97), with *P* < 0.05 for the two groups; there were 0 cases of urinary retention in the test group patients and 6 cases in the control group patients, with a statistically significant difference between the two groups, with *P* value < 0.05.

### 4.3. TRA Performed Cerebral Angiography Can Improve Patients' Comfort

Studies [2, 18] have shown that shortening bed rest and surgical limb braking time after total cerebral angiography helps improve patients' discomfort status and improve their postoperative hospital comfort, which greatly facilitates their recovery. The results of this pilot study showed that the test group was better than the control group in terms of GCQ scores (*P* value < 0.05), and the difference between the two groups was statistically significant.

Compared with the traditional transfemoral route, the success rate of puncture is relatively low, but it has the advantages of high safety, low postoperative bleeding complications, no combined application of active anticoagulation therapy, no bed rest, and shortened hospital stay, which are gradually being implemented in major hospitals [19, 20]. With the improvement of puncture technique and the popularization of medical devices, it has become one of the main ways of coronary angiography and interventional procedures [21, 22].

The main reasons for unsuccessful procedures are puncture failure and radial artery spasms. Multiple punctures can cause a loss of operator confidence and also lead to radial artery spasms [23, 24]. The highest failure rate of transradial artery surgery in small elderly women has been reported in the literature, which may be related to the small size of the radial artery and its susceptibility to spasms [25, 26]. Therefore, it is proposed that small elderly women are a relative contraindication to transradial artery surgery. In addition, the absence of radial artery pulsation, positive Allen's test, arteriovenous fistulae on renal dialysis, and treatment with sheaths of 8F or more are absolute contraindications. Patients with good radial artery pulsation and a negative Allen test should be selected.

Most of the operations are performed on the right side of the patient, using the right radial artery for puncture. In our department, the left pedal vein is mostly chosen as the venous access, and after two years of practice, it has been proved that the left pedal vein is superior to other parts of the venous access. The left pedal vein is far away from the surgical area, so changing the infusion does not affect the surgical operation. Intraoperative blood pressure monitoring also does not affect the infusion rate of the left foot vein.

Improving puncture technique and preventing radial artery spasms can improve the success rate of surgery. Preoperative elimination of patient tension, selection of patient-appropriate instruments, improvement of the first puncture success rate, injection of vasodilators via the radial artery, selection of small-sized catheters whenever possible, and gentle handling are all keys to successful surgery.

## 5. Conclusions

The rate of bleeding and urinary retention at the puncture site of transradial access puncture is lower than that of femoral access puncture during cerebral angiography, and the time to first urination of the patient after the procedure is significantly shorter, while the comfort of the patient after the procedure is improved to a greater extent, with excellent clinical results.

## Figures and Tables

**Table 1:** Comparison of general information between the two groups' cases (percentage, %).

Projects	Test group (*n* = 40)	Control group (*n* = 40)	Statistical values	*P*
Gender			0.808^2^	0.369
Male	20 (50)	24 (60)		
Female	20 (50)	16 (40)		
Age (years)	63.75 ± 8.51	62.67 ± 9.44	0.53^1^	0.594
Education level	—	—	0.115^2^	0.990
Elementary school and below	5 (12.5)	6 (15)		
Middle school				
High school or junior college	21 (52.5)	20 (50)		
College and above	6 (15)	6 (15)		
Marital status				
Unmarried	8 (20)	8 (20)		
Married			1.753^2^	0.416
Divorced or widowed	0 (0)	1 (2.5)		
Prothrombin time (sec)	32 (80)	34 (85)		
Platelets (10^9^/L)	8 (20)	5 (12.5)		
Duration of surgery (minutes)				

1-hour postoperative intake (ml)	11.56 ± 1.15	11.45 ± 1.28	−0.38^1^	0.702
	229.2 ± 41.67	241.3 ± 53.51	−1.13^1^	0.263

2-hour postoperative intake (ml)	38.47 ± 7.69	38.27 ± 7.50	0.12^1^	0.906
	243.8 ± 93.6	260 ± 103.7	−0.74^1^	0.464

4-hour postoperative intake (ml)	520.8 ± 132.2	504.3 ± 144.1	0.53^1^	0.595
	953.5 ± 198.6	965 ± 194.2	−0.26^1)^	0.794

*Note.* 1): *t*-value; 2)*χ*^2^-value.

**Table 2:** Comparison of postoperative puncture site bleeding, urinary retention, and GCQ scores between the two groups.

Group	Number of examples	Bleeding from puncture site with or without		First urination Time (minutes)	Urinary retention with or without		GCQ score
Test group	40	1 (2.5)	39 (97.5)	62.47 ± 15.24	0	40	70.65 ± 7.66

Control group	40	6 (15)	34 (85)	85.97 ± 32.88	6	34	61.45 ± 8.72

*χ* ^2^		3.914		−4.1^1^	6.486^2^		5.01^1^

*P*		0.048		0.0001	0.011		<0.0001

*Note.* 1): *t*-value; 2)*χ*^2^-value.

## Data Availability

The experimental data used to support the findings of this study are available from the corresponding author upon request.
